# Bioinformatics Analysis of the Characteristics and Correlation of m6A Methylation in Breast Cancer Progression

**DOI:** 10.1155/2022/4416439

**Published:** 2022-05-21

**Authors:** Ping Zhao, Xinwei Huang, Anhao Wu, Xin Yang, Yang Fu, Yuhang Quan, Ji Zhang, Zhen Li, Qi Tang, Maohua Wang

**Affiliations:** ^1^Department of Mammary Surgery I, The Third Affiliated Hospital of Kunming Medical University (Yunnan Cancer Hospital,Yunnan Cancer Center), Kunming 650118, China; ^2^Key Laboratory of the Second Affiliated Hospital of Kunming Medical University, Kunming 650101, China; ^3^Department of Blood Transfusion, The First People's Hospital of Yunnan Province, The Affiliated Hospital of Kunming University of Science and Technology, Kunming 650032, China; ^4^Department of Radiology, The First People's Hospital of Kunming, Kunming 650100, China; ^5^Department of Anesthesiology, The Third Affiliated Hospital of Kunming Medical University (Yunnan Cancer Hospital,Yunnan Cancer Center), Kunming 650118, China; ^6^Department of Mammary Surgery III, The Third Affiliated Hospital of Kunming Medical University (Yunnan Cancer Hospital,Yunnan Cancer Center), Kunming 650118, China; ^7^Department of Mammary Surgery II, The Third Affiliated Hospital of Kunming Medical University (Yunnan Cancer Hospital,Yunnan Cancer Center), Kunming 650118, China

## Abstract

Growing cutting-edge study has demonstrated the RNA m6A methylation's critical role in regulating tumorigenesis and progression all over the world, while it is still a mystery whether RNA m6A methylation has a positive impact on breast cancer treatment. In this article, we utilize bioinformatics to analyze three data sets including TCGA-BRCA, GSE96058, and GSE25066 and discover that breast cancer samples could be divided into 4 subtypes, which are quiescent, m6A methylation, protein-binding, and mixed, clarified by the expression level of m6A-related genes. R-survival analysis results also prove that the survival rate of breast cancer samples of the four subtypes significantly varies and remarkable differences in the number of exons' skip among the four subtypes can be seen according to the analysis of breast cancer gene expression characteristics. The degree of TP53 mutation and copy number loss is most obvious in the protein-binding subtype when it comes to tumor driver genes. Among the DNA damage repair genes, there is a sharp increase in the copy number of RAD54B of the protein-binding subtype, but fewer mutations in other DNA damage repair-related genes and copy number deletion is everywhere. Results of m6A methylation influencing on the proportion of infiltrated immune cells also indicate significant differences of the four m6A subgroups in macrophages M0 and mast cells resting which are closely correlated to patient prognosis. In addition, findings of the highest tumor stemness index and the lowest in the m6A methylated type in breast cancer samples can prove the critical role of the high expression of m6A reader protein in the progression of breast cancer.

## 1. Introduction

Breast cancer is the most common malignancy cancer of women all over the world. Globally, there are more than 1.7 million new cases occurring each year, with an increasing rate of 3 to 4 percent per year [1, 2]. Gene mutation and abnormal expression are important reasons for the occurrence and progression of breast cancer [3]. Studies have shown that each stage of tumor occurrence and progression is accompanied by changes in genetic information [4]. Compared with the lower frequency of gene mutation, the frequency of epigenetic modification changes is greatly increased [5]. Epigenetic modifications leading to changes in gene expression are common in tumor cells. Among them, the abnormal modification of RNA plays a key role in tumor progression. RNA modifications include 5-methylcytosine (m5C), pseudouridine, 2′-O-methylation, N1-methyladenosine (m1A), N7-methyladenosine and N6-methyladenosine (m6A), and so on [6]. Among these modifications, RNA m6A methylation is considered to be the most significant and abundant modification form in eukaryotic cells, and its abundance accounts for 0.1–0.4% of total adenosine residues [7]. The fat-mass and fat-associated protein is reported since 2011; the study on m6A methylation in tumors has attracted extensive attention [8].

M6A modification is a reversible process dynamically regulated by methyltransferases (“writers”), binding proteins (“readers”), and demethylases (“erasers”) [9, 10]. M6A methylation-related proteins are usually abnormally expressed in a variety of human cancer tissues, which in turn leads to abnormal expression levels of cancer-driving or tumor suppressor genes [11]. For example, YTHDF2 promotes the stem cell phenotype and tumor metastasis of hepatocellular carcinoma by recognizing the m6A methylated 5′-UTR of OCT4 mRNA [12]. M6A reader YTHDF1 promotes ovarian cancer progression by increasing EIF3C translation [13]. METTL3 protein and mRNA levels are highly expressed in pancreatic cancer tissues and cancer cells, and high METTL3 expression is associated with high N stage and pathological stage [14]. Abnormal expression of m6A-related proteins has a similar effect in breast cancer. M6A demethylase FTO promotes breast tumor progression by inhibiting BNIP3 expression [15]. In the hypoxic microenvironment, ALKBH5 is highly expressed in breast cancer, leading to the demethylation of m6A on NANOG mRNA and increasing the stability of NANOG mRNA, which promotes the enrichment of breast tumor stem cells [16]. In addition, it has been reported that the abnormal expression of m6A-related genes is related to the prognosis and survival of breast cancer patients. For example, the upregulated expression of YTHDF1, YTHDF3, and KIAA1429 is related to the poor prognosis of breast cancer [17]. The increase or decrease of m6A modification shows different results in different tumors. It has been previously reported that the mechanism of m6A modification in promoting cancer depends on the expression of m6A methylation-related proteins [18]. Therefore, breast cancer is divided into several subtypes according to the expression pattern of m6A methylation-related genes. At present, the relationship between the abnormal expression of m6A-related genes and clinical outcomes in patients is not clear, and the effect of m6A-related factors on the molecular characteristics of breast cancer has not been systematically reported [19]. In this study, the relationship between different m6A subtypes and survival, prognosis, mutation, copy number variation, immune cell infiltration, drug sensitivity, and tumor stemness index in breast cancer samples is analyzed.

## 2. Data and Methods

### 2.1. Data Collection

The data of this study are from TCGA and GEO, respectively, TCGA-BRCA, GSE96058 and GSE25066. The transcriptome data of the TCGA-BRCA dataset consisted of 1,217 samples, including 1,104 sequenced tumor tissue samples. The GSE96058 data set contains 3409 sequenced samples, including 136 biological replicate samples. The GSE25066 data set contains 508 samples. ComBat (SVA package, V3.36.0) and RUV Seq (V1.22.0) are used for batch effect removal [20]. Two different standardized algorithms, RUVr and RUVg, are used to remove batch effects.

### 2.2. M6A Gene Grouping and m6A Subtype Classification of Breast Cancer

The m6A gene set contains 8 writer genes (METTL15, METL15, RBM3, RBM15B, WTAP, CBLL1, KIAA1429, and ZC3H13), 2 eraser genes (ALKBH5 and FTO), and 11 reader genes (YTHDC1, YTHDC2, IGF2BP1, YTHDF1, YTHDF2, YTHDF3, HRNPA2B1, HNRNPC, FMR1, LRPPRC, and ELAVL1). According to the biological function, m6A-related genes are divided into two groups: Set1 (writer + reader) and Set2 (eraser). According to the *Z*-score median of Set1 and Set2 gene expression of the sample, the samples is divided into 4 types. They are static quiescent (setl≤0, set2≤0), m6A methylation (set1>0, set2≤0), protein binding (set1≤0, set2>0), and mixed (set1>0, set2>0).

### 2.3. Analysis of the Prognosis and Clinicopathological Indicators of the Four m6A Subtypes of Breast Cancer

The survival package of R is used to analyze the prognosis of the four m6A subtypes of breast cancer, and Circos is used to analyze the correlation between the four m6A subtypes of breast cancer and different clinicopathological indicators.

### 2.4. Analysis of Variable Splicing, Mutation, and Copy Number Variation of Four Breast Cancer m6A Subtypes

The alternative splicing data of the TCGA dataset is downloaded from TCGA SpliceSeq; 7 types of alternative splicing are provided by the database: Alternate Promoter (AP), Exon Skip (ES), Retained Intron (RD), Alternate Terminator (AT), Mutually Exclusive Exons (ME), Alternate Donor site (AD), and Alternate Acceptor site (AA). The download parameters are set to the following: percentage of samples with PSI value = 0, minimum PSI range (delta across samples) = 0, and minimum PSI standard deviation = 0. Percentage of samples with PSI value = 0.75 is used to filter PSI data [21]. The MSigDB database (V7.1) is used to download the gene annotation data of genes annotated by the GO term GO: 0006281. The R package Maftools is used to extract the top 10 genes with the most mutations in the TCGA-BRCA dataset and GO:0006281, as well as the mutation type and copy number mutation type information of these 20 genes. Heat maps are used to show the distribution of mutations and copy number variations of the top 10 tumor driver genes and DNA damage repair genes in the four m6A subtypes.

### 2.5. Analysis of Infiltrated Immune Cell and Immune Efficacy of Four Breast Cancer m6A Subtypes

Cibersort (V1.01) is used to analyze the proportion of immune cells in the four subtypes of tumor samples [22]. The coxph function in the survival (V3.2-3) package of R is used in the univariate cox analysis of the proportion of 22 immune cells to obtain the immune cell infiltration types that are significantly related to the prognosis of the four m6A subtypes of breast cancer. Meanwhile, the proportions of 22 immune cells in the four m6A subtypes of breast cancer are analyzed by ANOVA. The infiltration types of immune cells in the four m6A subtypes of breast cancer are obtained. Multivariate cox analysis is performed using the covariance of the immune infiltration ratio of different immune cells calculated by Cibersort, and the sum of the value multiplied by the corresponding immune infiltration ratio is used as the sample risk score. TIDE is used to analyze the differences in immune efficacy of the four m6A subtypes in the TCGA-BRCA and GES96058 data sets. The analysis is performed using the TIDE (https:/github.com/liulab-dfci/TIDEpy) default parameter [23].

### 2.6. Analysis of the Sensitivity Difference of Four m6A Subtypes with Anthracyclines

According to the method described in 1.2, breast cancer samples of GSE25066 are divided into 4 m6A types. Twelve m6A-related genes are used for sample typing: Set1 (FTO, WTAP, METTL3, RBM15B, and ZC3H13), Set2 (HNRNPA2B1, HNRNPC, ELAVL1, YTHDC1, LRPPRC, FMR1, and YTHDC2). In addition, based on the clinical data from the GSE25066 dataset, the sensitive and nonsensitive samples of the anthracyclines are extracted. The differences in the number of drug-sensitive and nonsensitive samples among the four m6A subtypes of breast cancer are compared.

### 2.7. Analysis of the Stemness Index of the Four m6A Subtypes of Breast Cancer

According to the mRNAsi value of TCGA-BRCA samples, the *t*-test is used to analyze the difference in mRNAsi dryness index among the 4 m6A subtypes. Cell stemness index mRNAsi is downloaded from PMID 29625051 [24].

### 2.8. Statistical Analysis

R (V4.0) is used for statistical tests. ANOVA or *t*-test is used to analyze the differences among different m6A subtypes. *p* value < 0.05 is considered statistically significant.

## 3. Experimental Result

### 3.1. Breast Cancer Typing Results Based on the Expression Level of m6A-Related Genes

To explore the m6A-related genes in breast cancer, the ComBat (SVA package, V3.36.0) and RUVSeq (V1.22.0) are used to remove batch effects between TCGA and GSE data sets. Then, the *Z*-score of TCGA and GSE data sets is extracted. The expression levels of m6A-related genes are firstly standardized by *Z*-score. Then, breast cancer samples are divided into four subtypes according to the *Z*-score median of m6A-related genes expression level in the samples in Set1 and Set2, as shown in Figure 1(a). The sample sizes of the four m6A methylation subtypes show similar distributions (proportions) in each data set, which indicate that the typing results of breast cancer samples based on the expression levels of m6A-related genes have good consistency in different data sets. In addition, the expression levels of 21 m6A methylation-related genes in four m6A subtype breast cancer samples are shown in Figure 1(b).

### 3.2. Analysis of Prognosis and Clinical Pathological Features of 4 m6A Breast Cancer Subtypes

The results of survival analysis show that there are significant prognostic differences among the 4 subtypes, as shown in Figure 2(a). Among them, the survival rate of mixed subtype samples is higher than that of the other three subtypes. In the triple-negative breast cancer samples, the survival of the four subtypes of breast cancer samples has more significant differences, as shown in Figure 2(b). In addition, the analysis results between m6A subtypes and clinical pathological features show that there is a significant quantitative difference between the m6A methylated subtypes and protein-binding subtypes of ER+. However, there are no significant differences among the four m6A subtypes in HER+/-, TNM staging, and age, as shown in Figure 2(c).

### 3.3. Analysis of Variable Splicing, Mutation, and Copy Number Variation of Four m6A Breast Cancer Subtypes

According to the statistical results of TCGA SpliceSeq, we find that there are differences in the number of ES between the four m6A subtypes, and the other six alternative splicing subtypes have no significant changes among the four m6A subtypes, as shown in Figure 3(a). Furthermore, the effect of the number of ES type on the prognosis of the four m6A subtypes is analyzed, and the results show that the m6A methylated subgroup is significantly different from the protein-bound subgroup in the prognosis, no matter in all samples or in triple-negative breast cancer samples, as shown in Figures 3(b) and 3(c). Next, the mutations and copy number variations of tumor driver factors and DNA damage repair genes of the four m6A subtype samples are analyzed. The 10 oncogenes with the most mutations in the TCGA-BRCA dataset are selected. The 10 genes were TTN, TP53, PIK3CA, CDH1, GATA3, KMT2C, MAP3K1, MUC16, RYR2, and HMCN1. The results show that TP53 was the gene with the most mutations and copy number loss in protein-binding type breast cancer samples, as shown in Figure 3(d). Moreover, the analysis of GO:0006281 gene set show that the 10 DNA damage repair genes with the most mutations are POLQ, TP53, BRCA2, ATRX, BRCA1, SETX, BLM, ATM, RAD54B, and ATR. Further analysis of the mutation types and copy number variation types of these 10 genes revealed that DNA damage repair genes are rarely mutated in breast cancer samples except for TP53. In terms of copy number variation, the copy number of RAD54B in the protein-bound subtype is increased, while the other 9 genes all show different degrees of copy number deletion in the 4 m6A subtypes, as shown in Figure 3(e).

### 3.4. Analysis of Immune Cell Infiltration in Four m6A Subtypes of Breast Cancer

Cibersort is used to analyze the types and proportions of infiltrated immune cells for TCGA and GSE96058 samples. The results show that a total of 22 types of immune cell infiltration, of which 11 types show significantly different infiltration rates among the 4 subgroups, as shown in Figure 4(a). Considering the influence of immune cell infiltration on the prognosis of the sample, univariate cox is performed to analyze the relationship between the proportion of immune cell infiltration and patient survival. The results indicate that the different proportion of NK cells resting and macrophages M0 leads to significant differences in patient survival time in all the samples, with HR < 1, as shown in Figure 4(b). In the triple-negative breast cancer samples, patient survival is significantly affected by the ratio of dendritic cell resting to mast cell resting, and HR < 1, as shown in Figure 4(c). Next, the types of immune cell infiltration with significant prognostic value in univariate cox analysis are demonstrated by multivariate prognostic analysis (risk value = proportion of immune cell infiltration ∗HR). The results show that NK cells resting and macrophages M0 are related to the survival of all samples in univariate prognostic analysis. The risk prediction results of high- and low-risk samples obtained by using the median risk value as the grouping index do not match the actual risk (risk value = *β* − NK cells resting × NK cells resting + *β* − macrophages M0 × macrophages M0), as shown in Figure 4(d). However, the multifactor risk prediction of dendritic cells resting and mast cells resting shows good risk prediction effects for triple-negative breast cancer samples, as shown in Figure 4(e). Based on the above analysis, mast cells resting and macrophages M0 is taken as the follow-up research object because of the significant differences between the two types of immune cell infiltration in the m6A subgroup, which also shows significant influence on the prognosis in univariate cox analysis. Further survival analysis reveals that the survival of all breast cancer samples is related to changes in the proportion of macrophages M0, as shown in Figure 4(f). Meanwhile, mast cells resting with significant prognostic value in triple-negative breast cancer is analyzed, as shown in Figure 4(g).

### 3.5. Differences in Immune Efficacy and Sensitivity to Anthracycline among the 4 m6A Subtypes

TIDE is used as an indicator of differences in immune efficacy. The results show that there is no significant difference in TIDE between the resting group and the m6A methylation group, as well as the mixed type and the m6A methylation group, and there are significant differences in immune efficacy between the other groups, as shown in Figure 5(a). Based on the grouping results of GSE25066 samples, the number of anthracyclines resistance and sensitivity samples of the 4 m6A subtype groups are compared. The results show that the number of drug-sensitive samples in the resting group is the least among the 4 subtypes. This result indicates that the expression of m6A gene contributed to the response of breast cancer to anthracyclines, as shown in Figure 5(b).

### 3.6. Differences in Stemness Index (mRNAsi) among the 4 m6A Subtype Groups

The higher the stemness index, the stronger the progression of the tumor. Elevated stemness promotes the progression of malignant behaviors of tumor cells, such as rapid and durable self-renewal, poor differentiation, and high malignancy. Our analysis results show that there is no significant difference in the stemness index between mixed and protein-bonding breast cancer samples. There are significant differences in tumor stemness index between breast cancer samples of other m6A subtypes. Specifically, the stemness index of the four subtypes of tumor samples from low to high are protein-bonding, mixed, quiescent, and m6A methylated, as shown in Figure 6. This result suggests that the expression of m6A writer and eraser alone will not lead to the increase of tumor stemness, while the expression of m6A reader is related to the increase of tumor cell stemness. In addition, the reason why the dryness index of resting breast cancer samples is higher than that of m6A methylated samples may be due to non-m6A factors.

## 4. Discussion

Based on the expression level of m6A in breast cancer, this study takes multiplatform and diverse data as the object, and the breast cancer samples are divided into 4 m6A subtypes according to the expression level of m6A. The results of this analysis indicate that m6A has important application value in the prognosis, detection of tumor progression, evaluation of chemotherapy effect and risk prediction of breast cancer patients, and m6A could be a new reference standard for the evaluation of breast cancer progression and prognosis. The formation process of m6A methylation is catalyzed by methyltransferases composed of WTAP, RBM15, METTL3, ZC3H13, METTL14, and KIAA1429, while the removal process is mediated by demethylases such as FTO and ALKBH5 [25]. M6A methylation level is related to the expression of methyltransferase and demethylase in cells. In addition, a group of specific RNA-binding proteins consisting of FMR1, HNRNPA2B1, LRPRC, YTHDF1/2/3, YTHDC1/2, and so on are necessary for m6A modification to exert effects [26]. The binding protein of m6A is a “double-edged sword”, which can not only promote the translation of mRNA, but also reduce the stability and accelerate degradation of mRNA [27]. More and more evidences indicate that the dysregulation of m6A regulatory factor is a key factor in the development of tumor.

In this study, differences in clinicopathological indicators, gene mutations, copy number variations, types and proportions of immune cell infiltration, immune efficacy, chemotherapeutic drug sensitivity, and tumor stemness are analyzed among the four m6A subtypes. Specifically, among the four breast cancer subtypes, the survival rate of the protein-binding subtype samples is significantly lower than the other samples. It has been shown that the decreased expression of m6A methylase (METTL3, METTL14, and WTAP) and the increased expression of m6A methylase (FTO and ALKBH5) in breast cancer are closely related to the progression and poor survival rate of breast cancer [28]. The upregulated expressions of m6A readers YTHDF1 and YTHDF3 are associated with metastasis and poor prognosis in breast cancer [27]. High expression of m6A binding protein has also been reported to be associated with poor prognosis and reduced survival of patients in other tumors except breast cancer. For instance, highly expressed LRPPRC is an effective marker for shorter BCP-free survival and OS in patients with metastatic PCa after androgen deprivation therapy [29–31]. These results indicate that the high expression of m6A-related proteins is an important factor for poor prognosis of tumors especially the m6A binding proteins. In terms of molecular characteristics, TP53 mutations and copy number loss are most common in protein-bound breast cancer samples. It is known that abnormal expression of m6A-related proteins regulates the expression of p53 by changing m6A modification levels. It is reported that the upregulated expression of YTHDF1 and HNRNPA2B1 in melanoma results in the inhibition of p53 expression [32–35]. However, the regulatory effect of TP53 on m6A-related protein expression has not been reported. We hypothesize that the mutation and copy number loss of TP53, a key tumor suppressor gene, reduce the inhibition of tumor suppressor genes, which could be the key to promoting the upregulation of m6A binding protein in breast cancer. It is confirmed that the expression of m6A binding protein IGF2BP1 mRNA is increased by 100 times in the study of fibrolamellar hepatocellular carcinoma, while the p53 cancer-suppressing pathway is significantly inactivated in the FL-HCC cells [36–38]. In addition, CNV deletions of DNA damage repair genes increase genomic instability, which is also an important factor for abnormal expression of m6A-related genes.

Considering the influence of the proportion and type of infiltrating immune cells on the prognosis of the sample, m6A gene expression and the proportion and subtypes of infiltrating immune cells are analyzed. The results reveal that the proportion of NK cells and macrophages M0 is significantly different in the 4 m6A subtypes and related to the patient survival time. However, in triple-negative breast cancer samples, the ratio of dendritic cells resting and mast cells resting are the main factors for the significant difference in survival time of the four m6A subtype samples. In fact, abnormal expression of m6A-related factors determines the type and proportion of infiltrating immune cells. For example, the infiltration of CD8+T cells in pancreatic cancer is reduced by the increase and loss of ALKBH5 at arm-level [39]. High expression of WTAP reduces tumor-associated T lymphocyte infiltration and immune response, leading to poor prognosis of gastric cancer [40]. In addition, this study reveals that the immune efficacy of m6A protein-binding breast cancer is significantly lower than that of other subtypes. This approach of predicting tumor therapy based on m6A-related factor expression has also been demonstrated in other tumor species. For example, glioma patients are divided into high-risk and low-risk groups according to the expression of m6A regulatory factor, and a good predictive effect is obtained in terms of prognosis and treatment effect [41]. In the comparison of chemotherapy resistance, the most chemotherapy-sensitive samples are protein-binding subtype breast cancer, while quiescent subtype has the least chemotherapy-sensitive samples. Similar studies have yielded different results in different tumors. Similarly, high expression of METTL3, YTHDF3, and YTHDF1 induced NSCLC drug resistance and metastasis by promoting m6A methylation of YAP mRNA and translating [42]. Finally, the analysis of tumor stemness shows that the m6A protein-binding breast cancer samples have the strongest tumor stemness among the four subtypes, which is consistent with the previous analysis.

## 5. Conclusion

The effects of different m6A-related factor expression levels on the prognosis, mutation, immunity, and chemotherapy of breast cancer samples are systematically and comprehensively analyzed. This result has positive significance for understanding the role of m6A molecular events in breast cancer, which may provide an important reference for the clinical treatment and prevention of breast cancer. The highest tumor stemness index and the lowest in the m6A methylated type in breast cancer samples can prove the critical role of the high expression of m6A reader protein in the progression of breast cancer.

## Figures and Tables

**Figure 1:** The expression levels of m6A-related genes in the four m6A subtype samples of breast cancer. (a) Based on the *Z*-score of m6A gene expression level, the expression differences of different m6A gene sets among the four breast cancer subtypes are shown. (b) Based on the *Z*-score of the m6A gene expression level, the expression differences of different m6A gene sets among the four subtypes were demonstrated.

**Figure 2:** Correlation analysis of prognosis and clinicopathological indicators of four m6A breast cancer subtypes. (a) Survival analysis of all samples. (b) Survival analysis of triple-negative breast cancer (TNBC) samples. (c) Correlation of four m6A breast cancer subtypes in TCGA-BRCA and GSE 96058 samples with clinicopathological indicators.

**Figure 3:** The differences of alternative splicing, mutation, and copy number variation in four m6A subtypes of breast cancer. (a) Statistics of the number of alternative splicing types in 4 m6A breast cancer subtype samples. (b) Survival analysis of m6A methylated subtype and protein-bound subtype in all breast cancer samples. (c) Survival analysis of m6A methylated subtype and protein-bound subtype in triple-negative breast cancer samples. (d) Differences in the number and type of tumor driver gene mutations and CNVS among the four m6A subtypes. (e) Differences in the number and type of DNA damage repair genes mutations and CNVS among the four m6A subtypes.

**Figure 4:** The effect of the types and proportions of infiltrating immune cells on the prognosis of the four m6A subtypes of breast cancer. (a) Types and proportions of immune cell infiltration in different breast cancer subtypes (ANOVA analysis). (b) Univariate COX is used to analyze the effect of immune cell infiltration ratio on the prognosis of breast cancer (all samples). (c) Univariate COX is used to analyze the effect of immune cell infiltration ratio on the prognosis of breast cancer (triple-negative breast cancer sample). (d) Multivariate prognostic analysis of NK cells resting and macrophages M0 in breast cancer samples. (e) Multivariate risk prediction of dendritic cells resting and mast cells resting in triple-negative breast cancer samples. (f) The difference in the proportion of infiltrated macrophages M0 in the prognosis of the four m6A subtypes of breast cancer (all samples). (g) The difference in the ratio of mast cell resting infiltration among the 4 m6A breast cancer subtypes (triple-negative breast cancer samples).

**Figure 5:** Differences in immune efficacy and sensitivity to anthracycline in 4 breast cancer subtypes of m6A. (a) Difference in immune response among four m6A subtypes (*t*-test). (b) Differences of resistance and sensitivity to taxane anthracycline of four m6A subtypes.

**Figure 6:** Differences in the tumor dry index between the four m6A subtypes.

## Data Availability

The simulation experiment data used to support the findings of this study are available from the corresponding author upon request.
